# Link between the aboveground and belowground biomass allocation with growing of *Tamarix* sp. seedlings in the hinterland of Taklimakan Desert, China

**DOI:** 10.1371/journal.pone.0289670

**Published:** 2023-08-16

**Authors:** Flora Erkin, Dai Yue, Anwar Abdureyim, Wanyuan Huang, Mawlida Tayir

**Affiliations:** 1 College of Ecology and Environment, Xinjiang University, Urumqi, China; 2 Key Laboratory of Oasis Ecology, Ministry of Education, Xinjiang University, Urumqi, China; 3 College of Geography and Remote Sensing Science, Xinjiang University, Urumqi, China; Ningbo University, CHINA

## Abstract

The morphological characteristics and biomass allocation can reflect plant adaptive strategies to the environment. *Tamarix* sp. is an excellent shrub species used for windbreaks and fixing sand in the desert of northwest China. The successful establishment of *Tamarix* sp. seedlings and their growth into mature individuals require their adaptation to various environmental conditions, which is the key to naturally regenerating the *Tamarix* population. To clarify the root morphological characteristics, leaf structural characters, and biomass allocation of *Tamarix* sp. seedlings in response to drought conditions, we took the *Tamarix* sp. seedlings at the Daryaboyi oasis in the hinterland of Taklimakan Desert as the object of study, analyzed rooting depth, root dry weight (RDW), specific root length (SRL), root surface area (RA), specific root area (SRA), leaf area (LA), specific leaf area (SLA) and root: shoot ratio (R:S ratio). The gravimetric soil water content varied from 5.80% to 25.84% in this study area. The taproots of *Tamarix* sp seedlings with small basal stem diameters were shallower and had few lateral root branches and *Tamarix* sp. seedlings with large basal stem diameters had more obvious taproots and lateral roots. With the growth of *Tamarix* sp. seedlings, the taproot deepened, and the values ranged from 4.5 cm to 108.0 cm; the SRL, SRA, and SLA decreased, and the ranges of the values were 28.92–478.79 cm·g^-1^, 1.07–458.50 cm^2^·g^-1^, and 24.48–50.7 cm^2^·g^-1^; the RDW, RA, and LA increased, the ranges of the values were 0.16–21.34 g, 3.42–328.04 cm^2^, and 2.41–694.45 cm^2^; the more biomass was allocated to the aboveground parts, and the mean R: S ratio was 0.76. In better soil water conditions, the root growth rate decreased as *Tamarix* sp. seedlings grew, and more biomass was allocated to the aboveground. This further showed that stable surface water is highly significant to the biomass allocation strategy of *Tamarix* sp. seedlings.

## 1 Introduction

The Taklamakan Desert is the largest desert in China and the second-largest mobile desert in the world. The ecological environment of the Taklamakan Desert is extremely harsh and the climate is dry ‎[1]. Therefore, some excellent drought-resistant and sand-fixing pioneer plants have become the dominant species here. *Tamarix* sp. is an excellent shrub in the desert of northwest China ‎[2]. It is often regarded as a pioneer plant for wind and sand control due to its excellent resistance to growth and reproduction in the harsh environment of desert areas and to influence and improve the desert environment through its rapid growth and development ‎[3, 4].

Plant functional traits indicate the ability of plants to grow, reproduce and survive by affecting plant growth, reproduction, and survivability and thus indirectly affecting its morphological and physiological traits [5]. Functional traits that help plants in acquiring limiting nutrients and water are more important for desert plant species ‎[6, 7]. The roots and leaves are important organs for energy and material exchange between plants and the environment. Root morphological characteristics are used as indicators of resource utilization strategies, which can reflect the adaptation and competitive ability of different species or provenances, to survive during the long-term evolutionary process ‎[8]. When plants are exposed to water stress, to maintain the absorption of water and nutrients, the roots of plants must enter the deep soil layer and continue to grow rapidly ‎[9]. Previous studies have found that under drought conditions the specific root length (SRL) decreased, root surface area (RA) and specific root area (SRA) increased ‎[10, 11], can conclude that plants can change their morphology through regulation, adapt to changes in environmental conditions, and increase the survival probability.

Plant leaf functional traits can not only reflect plant growth, metabolism, and reproduction but also represent plant adaptation strategies to different ecological environments ‎[12]. The leaf area (LA) is an important parameter to evaluate many traits of plants like canopy, photosynthesis, and evapotranspiration ‎[13, 14]. The specific leaf area (SLA) is defined as the light-capturing leaf surface area per unit of dry biomass ‎[15], and an essential functional trait and indicator for estimating plant strategies in response to environmental changes ‎[12]. Plant traits are often interdependent, or their values correlate, LA and SLA are informative on resource acquisition and lifespan ‎[16]. Plants adopt low LA and low SLA adaptation strategies to maintain water in an arid environment, whereas contrasting values are implying quick nutrient use and photosynthetic capacity ‎[17, 18]. In summary, LA and SLA are closely related to light availability and habitat resource supply.

The allocation of biomass to plant organs plays an important role in their acquisition of resources and competition to survive ‎[19]. Optimal partitioning theory (OPT) suggests that plants should allocate biomass to the organ that acquires the most limiting resource ‎[20]. Padilla et al. ‎[21] find that roots of all species responded to alterations in water supply by changing biomass allocation patterns (i.e., higher root: shoot ratio (R:S ratio) in droughted plants), and by altering fine roots diameter, measured in terms of SRL. When plants are stressed by water and nutrients, the biomass allocated to the roots increases to obtain more water and nutrients ‎[22]. Past few years studies found that under irrigation conditions, higher water and nutrients enable plants to allocate more biomass to the aboveground (i.e., R: S ratio decreased) ‎[3, 23, 24]. Meanwhile, it shows that the increase of the belowground part can mitigate the conditions when a plant’s supply is lower in nutrients and water ‎[25].

The Daryaboyi Oasis is located at the tail of the Keriya River, which is the second-largest river at the southern edge of the Tarim Basin. The oasis is subject to relatively little interference and thrives under natural conditions, with relatively "primitive" characteristics ‎[26]. *Tamarix* sp. (bush species) is one of the dominant species in the Daryaboyi oasis. The seedling stage is the most vulnerable stage during plant settlement and the stage at which the plants are most likely to die ‎[27]. The successful settlement and growth of *Tamarix* sp. seedlings into mature individuals need to adapt to various adverse conditions, which is the key to realizing the natural renewal of the *Tamarix* population. Recent years studies showed that the Daryaboyi Oasis has inundation from 2000 to 2019, with maximum peaks occurring in February and August; a period of minimal inundation occurred in May ‎[28, 29]. River water is a critical parameter for the germination and growth of *Tamarix* sp. seedlings in this study area. Currently, studies on root morphological characteristics, leaf structural characters, and biomass allocation have focused on adult *Tamarix* sp. in plantations ‎[30–32]. While less attention has been paid to these characteristics in *Tamarix* sp. seedlings grown under natural environmental conditions. Therefore, in this study, we analyzed the root morphological characteristics, leaf structural characters, and biomass allocation of *Tamarix* sp. seedlings during their early growth stages, which is important to help improve the understanding of the mechanisms used by plants to adapt to arid zones. Therefore, two specific hypotheses were tested: In a natural environment with perennial surface water runoff, with the growing of *Tamarix* sp. seedlings in the hinterland of Taklimakan Desert (1) they decrease SRA and SLA, and (2) allocated more biomass to the aboveground.

## 2 Materials and methods

### 2.1 Study area

The study area is located at the Daryaboyi Oasis in the hinterland of the Taklamakan Desert, Xinjiang, China (Fig 1). It has a geographical location of 38°24’–38°34’N, 81°56’–81°90’E, an altitude of 1,100–1,300 m, and an area of approximately 324 km^2^ ‎[33, 34]. This area is part of a typically arid continental climate, with an average annual precipitation of less than 10 mm; the average relative humidity is 40.2%; the annual potential evaporation is 2,480 mm; the average annual temperature is 12.1°C, and there is a large difference in temperature between day and night ‎[22]. The primary plant species in the oasis are *Populus euphratica* Olivier, *Tamarix* spp., *Alhagi sparsifolia* Shap, *Phragmites australis* (Cav.) Trin ex. Steud, and *Karelinia caspia* Less. The depth of the groundwater table ranges from 1 to 8 m in the oasis from south to north; the winter and spring seasons have shallower groundwater depth than the summer and autumn seasons ‎[26]. The annual river runoff is relatively stable, with a large amount from September to February and a small amount from March to August ‎[35]. The soil is primarily sandy, and the concentrations of soil organic carbon (SOC) and total nitrogen (TN) are 2.14 g·kg^-1^ and 0.08 g·kg^-1^ respectively. The pH value of the soil is 9.22.

**Fig 1:** Location of the study site.

### 2.2 Experimental design

We conducted field sampling after obtaining permission from the government of Daryaboyi Township, Yutian County, Hotan Region, Xinjiang, China. The field experiment was conducted in mid-June 2021. There was surface runoff in the sampling area in early June 2021, and the groundwater depth was 2.40 m. Representative areas of *Tamarix* sp. seedlings were selected that were subject to less human interference and near the established groundwater observation wells in the oasis, and samples of their leaves, roots, and nearby soil were collected. We randomly selected three sample plots (1 × 1 m) near the observation well, and the height, crown width, basal stem diameter, and coverage of *Tamarix* sp. seedlings in the sample plots were measured, and the average values were 22.8±16.0 cm, 11.6±7.1 cm, 4.9±2.5 mm, and 30.45%, respectively.

### 2.3 Sampling and measurements

#### 2.3.1 Plant sampling

Growing well, free of insects and diseases, and had a representative basal stem diameter *Tamarix* sp. seedlings that ranged from 1 to 11 mm were randomly selected from the sample plots. The whole roots of 12 *Tamarix* sp. seedlings were excavated in the sample plot, and their morphological information is shown in Table 1, and the list of root and leaf functional traits, their abbreviations, and definition are shown in Table 2. Tools, such as shovels, tweezers, brushes, and thin wooden sticks, were used to carefully strip away the soil around the roots until they were fully exposed. We maintain the integrity of the root system during the excavation. If there were broken roots, the roots were labeled. The position of their growth was recorded, and the roots were photographed for measuring RA and SRA. The roots were separated from the aboveground parts and placed in numbered airtight bags. The aboveground part of the *Tamarix* sp. seedlings to determine the R: S ratio, and leaves were photographed for measuring LA and SLA

**Table 1:** Morphological information of the whole roots excavated from *Tamarix* sp. seedlings (means ± SD).

Basal stem diameter (mm)	Plant height (cm)	Crown width (cm)	Rooting depth (cm)	Sample number
0–2	4.08±0.80	3.73±0.61	37.17±23.13	3
2–5	11.40±0.28	6.38±3.65	62.5±17.78	3
5–11	35.42±5.30	37.9±7.21	67.25±18.89	6

**Table 2:** List of root and leaf functional traits and their abbreviations.

Traits	Abbreviations	Unit	Ecological significance and references
Root dry weight	RDW	g	a structural material, which can reflect the vitality and quality of roots ‎[36].
Specific root length	SRL	cm·g-1	the ratio of root length to biomass, which can represent the relationship between root gain and expenditure ‎[37].
Root surface area	RA	cm2	reflect the effective absorption area of water and nutrients absorbed by roots as a whole ‎[38].
Specific root area	SRA	cm·g-2	represents the ability to exchange
			processes between the roots and soil ‎[39].
Leaf area	LA	cm2	the important parameter to evaluate many traits of plants like canopy, photosynthesis, and evapotranspiration ‎[13, 40].
Specific leaf area	SLA	cm·g-2	plays an important role in determining the productivity of plants ‎[41].
Root: shoot ratio	R: S	/	reflects many internal basic changes and the process of self-adaptation and self-adjustment under the effect of environmental factors ‎[3].

The calculation formula for the R: S ratio is as follows ‎[3]


$$R:S\;ratio=\frac{{DW}_{belowground}}{{DW}_{aboveground}}$$ (1)

Where the DW_belowground_ is the dry weight of belowground biomass, and DW_aboveground_ is the dry weight of aboveground biomass.

All the leaves and roots on the full-root excavation plant were placed on different white papers with references and photographed. Adobe Photoshop 2020 (Adobe, San Diego, CA, USA) was used for cutout graphics (Fig 3). The calculate leaf and root area software (HP Scan jet 4850) was used to calculate the surface areas of leaves and roots. The leaves and roots were then placed in a 60°C oven for 48 h to determine the constant weight to calculate the SRL, SRA, and SLA. The formulae are as follows ‎[37, 39, 41]:

$$\mathrm{SRL}=\frac{RL}{RW}$$ (2)

$$\mathrm{SRA}=\frac{RA}{RDW}$$ (3)

$$\mathrm{SLA}=\frac{LA}{LW}$$ (4)

Where SRL is the specific root length; RL is the total root length (cm), and RDW is the total root dry weight (g). SRA is the specific root area; RA is the total root area (cm^2^); SLA is the specific leaf area; LA is the single leaf area (cm^2^), and LW is the leaf dry weight (g).

#### 2.3.2 Soil sampling

The soil samples were collected at intervals of 20 cm near the plants sampling plants from the topsoil to the groundwater table, and there were three replicates per layer. The soil sample was placed in an aluminum box and brought back to the laboratory to measure the gravimetric soil water content (SWC) by oven drying method. Other soil samples were simultaneously taken from the 0–20 cm layer in the sample plot and placed in sealed bags for numbering, which was used to determine the SOC, TN, TP, and pH value. The SOC was determined by the black dichromate oxidation method; the soil TN was measured by the semi-micro Kjeldahl digestion procedure; the soil TP was determined by spectrophotometry ‎[42]. To determine the soil pH, the electrometric method as described by Adams and Pearson ‎[40] was used.

The formula to calculate the SWC is as follows ‎[43]:

$$SWC=\frac{\left({FW}_{soil}-{DW}_{soil}\right)}{{DW}_{soil}}$$ (5)

Where SWC is the gravimetric soil water content; FW_soil_ is the fresh weight of soil, and DW_soil_ is the dry weight of soil.

### 2.4 Data analysis

All data were analyzed using SPSS 22.0 (SPSS Inc., China go, IL, USA). The relationships between basal stem diameter and RDW, SRL, RA, SRA, LA, and SLA, and that between Ln root mass and Ln shoot mass, and between R: S and Ln total mass were fitted via linear regression models by Origin 2021. All Graphs were plotted with Origin 2021.

## 3 Results

### 3.1 Characteristics of gravimetric soil water content

The SWC in the study area increased with the increase in soil depth (Fig 2). The SWC varied from 5.80% to 25.84%, with an average of 15.12%, and it fluctuated in the 0–120 cm soil depth, with a varied range of 5.80% to 19.49%. Below the 120 cm soil depth, the SWC gradually increased.

**Fig 2:** Variation of gravimetric soil water content at different depths at the Daryaboyi Oasis in the hinterland of the Taklimakan Desert, China (means ± SD, n = 3).

### 3.2 Root morphological characteristics and leaf structural characters of the *Tamarix* sp. seedlings

The root distribution of the *Tamarix* sp. seedlings varied with the size of the basal stem diameter (Fig 3). The taproots of *Tamarix* sp. seedlings with small basal stem diameters were obviously shallower and had few lateral root branches (Fig 3A and 3B). The taproots and lateral roots of *Tamarix* sp. seedlings with large basal stem diameters were more apparent (Fig 3C). The values of basal stem diameters were 1.40 mm, 2.95 mm, and 10.63 mm; the taproot lengths were 35.4 cm, 54.1 cm, and 31.8 cm, respectively, and the root depths were 52 cm, 54.1 cm, and 108 cm, respectively. The depth of *Tamarix* sp. seedling taproots deepened as the basal stem diameters increased, and the root depth varied from 4.5 cm to 108.0 cm (Fig 4).

**Fig 3:** Root distribution of *Tamarix* sp. seedlings with different basal stem diameters. Note: the basal stem diameters were as follows: (a) 1.40 mm, (b) 2.95 mm, (c) 10.63 mm.

**Fig 4:** Taproot depths of *Tamarix* sp. seedlings individual with different basal stem diameters.

The linear regression models of the RDW and RA of *Tamarix* sp. seedlings were *y* = 1.84*x*-4.64 and *y* = 10.27*x*+16.86 (Fig 5A and 5C), with the slope of RDW and RA vs. basal stem diameter significantly higher than 1.0, this indicates that with the increase in basal stem diameter the RDW and RA increased, the ranges of the values were 0.16–21.34 g and 3.42–328.04 cm^2^, and the mean values were 5.69 g and 76.30 cm^2^. Fig 5B and 5D showed that linear regression models of the SRL and SRA of *Tamarix* sp. seedlings were *y* = -21.57*x*+300.89 and *y* = -5.39*x*+66.64, this indicates that with the increase in basal stem diameter, the SRL and SRA decreased, and the ranges of the values were 28.92–478.79 cm·g^-1^ and 1.07–458.50 cm^2^·g^-1^, the mean values were 179.42 cm·g^-1^ and 67.55 cm^2^·g^-1^, respectively.

**Fig 5:** Root morphological characteristics of *Tamarix* sp. seedlings with different basal stem diameters. Note: (a) root dry weight, (b) specific root length, (c) root area, (d) and specific root area.

The linear regression of the LA and basal stem diameter was proportional (Fig 6A), and the linear regression model was *y* = 60.34*x*-115.86, this indicates that with the increase of basal stem diameter, the LA of *Tamarix* sp. seedlings increased, and the ranges of the values were 2.41–694.45 cm^2^ and the mean LA values were 223.98 cm^2^. The linear regression of the SLA and basal stem diameter was inversely proportional (Fig 6B), and the linear regression model was *y* = -0.62*x*+41.66, this indicates that with the increase of basal stem diameter, the SLA of *Tamarix* sp. seedlings decreased, and the ranges of the values were 24.48–50.7 cm^2^·g^-1^ and the mean SLA values were 38.19±7.34 cm^2^·g^-1^.

**Fig 6:** Leaf area (a) and leaf specific area (b) of *Tamarix* sp. seedlings with different basal stem diameters.

### 3.3 Biomass allocation of the *Tamarix* sp. seedlings

The natural logarithms of root biomass and shoot biomass were tightly and linearly correlated (Fig 7A), the natural logarithms function was *y* = 0.87*x*-0.3. Thus, Fig 7A indicates that with the increase in basal stem diameter, both the aboveground and belowground biomass of *Tamarix* sp. seedlings increased. The linear correlation (*y* = -0.6*x*+0.89) between the R: S ratio and total mass shows that the R: S ratio decreases gradually with the increase in basal stem diameter, and the average R: S ratio was 0.76 (Fig 7B).

**Fig 7:** Aboveground and belowground biomass allocation of *Tamarix* sp. seedlings with different basal stem diameters.

## 4 Discussion

In arid and semiarid areas, soil water is a key factor that restricts plant growth and reproduction, affects the development of individual plants, determines the types of plants, and limits the distribution of vegetation ‎[44]. In the Daryaboyi Oasis, the SWC increased as the soil depth deepened, which was consistent with the results of soil water research in the Taklimakan Desert ‎[45]. Wan et al. ‎[46] showed that the shallow soil water in the Daliyabuyi oasis of the Taklimakan Desert was less than 1% without surface water. In our study area, surface water flows through, so the shallow soil has a high content of water (Fig 2), which facilitated the survival and growth of seedlings with shallow roots.

In an arid desert environment, the common ecological mechanism of plant adaptation to drought is a highly developed root system, with a deeper root depth ‎‎[3, 47]. The root morphological characteristics were closely linked to the utilization of water and nutrient resources by the plant ‎[48, 49]. The vertical roots stopped growing when the SWC reached 30% ‎[50]. Our results showed that the lateral root distribution of the *Tamarix* sp. seedlings with larger basal stem diameters was more apparent (Fig 3). The rooting depth of *Tamarix* sp. seedlings with different basal stem diameters generally increased as the basal stem diameter increased (Fig 4), indicating that the *Tamarix* sp. seedlings as the growing developed roots and tended to absorb deeper stable soil water.

The interaction between water status and RDW, RA, and R: S ratio was significant, drought increased R: S ratio but it reduced the RA and RDW ‎[51]. The RDW and RA of *Tamarix* sp. seedlings increased as the basal stem diameter increased (Fig 5A and 5C), which means good water conditions in our study area. The SRL is the ratio of root length to biomass, which can represent the relationship between root gain and expenditure ‎[37, 52]. The results of previous studies showed that the SRL of the *Abies* community decreased with tree size and aboveground biomass, and the mean value of SRL was 10.40 ± 0.26 cm·g^-1^ ‎[53]. The mean SRL was 18.2 cm·g^-1^ of the rainforest vascular epiphyte community ‎[54]. With the growth, the SRL values of *Tamarix* sp. seedlings decreased, and the mean value of SRL was 179.42 cm·g^-1^ (Fig 5B), the SRL of *Tamarix* sp. seedlings in our study area was higher, indicating that the productivity of *Tamarix* sp. seedlings was higher. The SRL and RA ranged from 730–940 cm·g^-1^ and 6.3–12 cm^2^ of *Platycladus orientalis* seedlings in a greenhouse ‎[55]. The plants that grow more quickly generally have a larger SRL than the plants that grow more slowly ‎[56]. It is therefore understandable that the *Tamarix* sp. seedlings were at a rapid growth stage in our study. The RA can reflect the effective absorption area of water and nutrients absorbed by roots as a whole ‎[38]. Drought treatment promoted the elongation growth of the root and increased its SRL and SRA ‎[43]. In sandy soil substrate, the response of seedlings to deeper phreatic water depth is realized by the increase of RA caused by the increase of total root length ‎[38]. In our study, with the growth of *Tamarix* sp. seedlings, RA increased (Fig 5C), which indicated that the growing *Tamarix* sp. seedlings by increasing the RA to capture more water. The plant growth theory suggests that fast-growing plants generally have a larger SRA. Plants with a larger SRA are more efficient at absorbing higher amounts of water and nutrients ‎[57]. In this study, with the increase in basal stem diameter, the SRA of *Tamarix* sp. seedlings decreased (Fig 5D), and the seedlings with the smallest basal stem diameters had the largest SRA. We can conclude that seedlings with small basal stem diameters applied a substantial amount of photosynthetic products into developing root systems to acquire stable water sources, further showing that small seedlings need higher water and nutrients during rapid growth. For instance, the SRL and SRA of Chinese fir plantations decreased with stand age, indicating that the fine root nutrient foraging ability decreased in older stands ‎[58]. From the results of these previous studies, we can confirm that the root growth rate decreased as *Tamarix* sp. seedlings grew.

Many studies have proved that plants in the desert change leaf functional traits to reduce water loss ‎[59, 60]‎. A study on leaf functional traits of *Disanthus cercidifolius* var. longipes H. T. Chang in the high mountains of southeastern China showed that as the plants developed, the LA increased and SLA decreased ‎[14]. As the same, with the growth of the *Tamarix* sp. seedlings, the LA increased (Fig 6A) and SLA decreased (Fig 6B). The SLA plays an important role in determining the productivity of plants since the changes in leaf SLA reflect changes to the structure and nutritional content of leaves ‎[41]. Previous studies have shown that plants with a low SLA live in relatively arid and barren environments, while those with a high SLA have a high rate of relative growth and productivity ‎[61]. The mean SLA of adult *T*. *chinensis* at the pure stand, mixed forest in the hinterland of the Taklimakan desert was 39.06±6.87 cm^2^·g^-1^ ‎[59]. The mean SLA of *Tamarix* sp. seedlings was 38.19±7.34 cm^2^·g^-1^ (Fig 6B), the SLA values of adults and seedlings were similar, which indicated that the seedling productivity of *Tamarix* sp. reached the adult`s level. The value of SLA from the present study was lower than the mean SLA (53±2 cm^2^·g^-1^) of the Mediterranean plant genus growing in northeastern Spain ‎[62], which indicates that plants in habitats with abundant resources typically have higher SLA values than plants in the desert with scarce resources. When the environment was dry and resources were scarce, *Haloxylon ammodendron* in the Ebinur Lake wetland, in Xinjiang, China reduced its SLA ‎[63]. The combination of soil nutrients and changes in LA and SLA of *Tamarix* sp. seedlings can be understood that the habitat soil is infertile.

Previous studies have shown that with the increase of drought, plants show strong drought resistance through root growth, SRL, RA, and SRA increasing ‎[43]. Compared with the decreasing trend of SRL and SRA as the growth of *Tamarix* sp. seedlings, and SLA reflected a low fitting slope, which indicates that the stability of photosynthetic function is maintained. In conclusion, the morphological characteristics of *Tamarix* sp. seedlings did not show drought-resistant properties, since the study area had good soil water conditions. This indicates that the conclusions were consistent with our hypothesis (1) that in a natural environment with perennial surface water runoff, with the growing of *Tamarix* sp. seedlings in the hinterland of Taklimakan Desert, they decrease SRA and SLA.

The increase in the R: S ratio enlarges the quantity of water and nutrients that is absorbed and enhances the ability of plants to resist drought and remain fertile ‎[3, 64]‎. When irrigation was timed roughly to coincide with local flooding the biomass of *Tamarix* sp. seedlings was primarily distributed to the aboveground parts, and the mean R: S ratio was 0.75 ‎[65], which was very close to the R: S ratio change trend of *Tamarix* sp. seedlings in this study (Fig 7A) and the average value of 0.76 (Fig 7). The response of *H*. *ammodendron* seedlings in the hinterland of the Taklamakan Desert in China to irrigation amount showed that the R:S ratio increased with decreasing irrigation amount and the R:S ratio was 0.92 when irrigation was minimal ‎[66]. Compare with the above study the small R: S ratio of *Tamarix* sp. seedlings indicated that the soil water condition was well in the study area, and more biomass was then allocated to the aboveground parts of the *Tamarix* sp. seedlings (Fig 7B). This indicates that the conclusions were consistent with our hypothesis (2) that under natural conditions, with the growth of *Tamarix* sp. seedlings in the hinterland of Taklimakan Desert allocated more biomass to the aboveground.

## 5 Conclusion

The study area was nourished by surface water from the Keriya River, the groundwater was shallow. The taproots of *Tamarix* sp. seedlings with small basal stem diameters were shallower and had few lateral root branches and *Tamarix* sp. seedlings with large basal stem diameters have more obvious taproots and lateral roots. Because the soil water condition is well, with the growth of *Tamarix* sp. seedlings, the root dry weight and root surface area increased, and the specific root length was higher, which indicated that *Tamarix* sp. seedlings have higher productivity and were at a rapid growth stage. The seedlings with the small basal stem diameters had the largest specific root area, can understand that small seedlings need higher water and nutrients during rapid growth. From the above results, it is clear that the root growth rate decreased as *Tamarix* sp. seedlings grew. The root: shoot ratio mean value was 0.76, and more biomass was allocated to aboveground parts with the growth of *Tamarix* sp. seedlings. This further showed that stable surface water is highly significant to the biomass allocation strategy of *Tamarix* sp. seedlings.
